The article "Knockdown of STIM1 expression inhibits non-small-cell lung cancer cell proliferation in vitro and in nude mouse xenografts" was published in 2019. Journal: Bioengineered.

# Knockdown of STIM1 expression inhibits non-small-cell lung cancer cell proliferation *in vitro* and in nude mouse xenografts

**DOI:** 10.1080/21655979.2019.1669518

**Published:** 2019-09-28

**Authors:** Chunlei Ge, Baozhen Zeng, Ruilei Li, Zhen Li, Qiaofen Fu, Weiwei Wang, Zhenyu Wang, Suwei Dong, Zhangchao Lai, Ying Wang, Yuanbo Xue, Jiyin Guo, Tiannan Di, Xin Song

**Affiliations:** a Department of Cancer Biotherapy Center, The Third Affiliated Hospital of Kunming Medical University (Tumor Hospital of Yunnan Province), Kunming, Yunnan, China; b Department of Thoracic Surgery, The Third Affiliated Hospital of Kunming Medical University (Tumor Hospital of Yunnan Province), Kunming, Yunnan, China; c Department of Biomedical Engineering Research Center, Kunming Medical University, Kunming, Yunnan, China

**Keywords:** Non-small-cell lung cancer, stromal interaction molecule 1, immunohistochemistry, cell cycle, proliferation

## Abstract

Stromal interaction molecule 1 (STIM1) is a calcium-sensing protein localized in the membrane of the endoplasmic reticulum. The expression of STIM1 has been shown to be closely associated with cell proliferation. The aim of the present study was to investigate the role of STIM1 in the regulation of cancer progression and its clinical relevance. The data demonstrated that the expression of the STIM1 was significantly higher in non-small-cell lung cancer (NSCLC) tissues than in benign lesions and was associated with advanced NSCLC T stage. Knockdown of STIM1 expression in NSCLC cell lines A549 and SK-MES-1 significantly inhibited cell proliferation and induces A549 and SK-MES-1 cell arrest at the G2/M and S phases of the cell cycle. Western blotting showed that the expression of cyclin-dependent kinase (CDK) 1 and CDK2 were reduced while knockdown of STIM1 expression. Furthermore, knockdown of STIM1 in NSCLC cells significantly reduced the levels of xenograft tumor growth in nude mice. These data indicate that aberrant expression of the STIM1 protein may contribute to NSCLC progression. Future studies should focus on targeting STIM1 as a novel strategy for NSCLC therapy.

## Introduction

Lung cancer is the leading cause of cancer-related mortality in both men and women worldwide [1]. Histologically, non-small-cell lung cancer (NSCLC) accounts for ~80% of lung cancer cases and is a heterogeneous clinical entity with the major histological subtypes comprising squamous cell carcinoma, adenocarcinoma and large-cell carcinoma [2]. The overall 5-year survival remains of NSCLC is poor, and evenfor patients with early-stage disease who undergocuratively intended surgery, the postoperative recur-rence rate is high compared to other types of cancer [3]. Therefore, there is an urgent need to study the underlying pathogenesis to enable early detection and prevention of lung cancer, and to identify new therapeutic targets for NSCLC.

The article "Knockdown of STIM1 expression inhibits non-small-cell lung cancer cell proliferation in vitro and in nude mouse xenografts" was published in 2019. Journal: Bioengineered.

With the identification of the molecular processes involved in pulmonary carcinogenesis, novel treatments targeting small molecules have emerged with encouraging results. For example, Ca^2+^ signaling controls a wide variety of cell functions, such as secretion, gene transcription, cell proliferation and apoptosis [4–6]. Alterations of Ca^2+^ signaling have emerged to an important factor in cancer progression [7,8]. Store-operated calcium entry (SOCE), a major Ca^2+^ influx mechanism activated upon Ca_2+_ storage depletion, is a ubiquitous mechanism for Ca^2+^ influx in non-excitable cells [9], while stromal interaction molecule 1 (STIM1) is a calcium sensor predominantly localized in the endoplasmic reticulum (ER). STIM1 interacts with Orail, which is identified as the major store-operated Ca^2+^  channel (SOC) in the plasma membrane, and initiate SOCE and refill of intracellular Ca^2+^ stores [10].

Moreover, STIM1 was identified and mapped to chromosome 11p15.5 in 1995 [11]. The STIM1 protein is a highly conserved type-I membrane protein containing a luminal EF-hand Ca^2+^ binding domain and several cytosolic protein-protein interaction domains [12,13]. Although the function of STIM1-SOCE has been well characterized in non-excitable cells, the role of STIM1 in the regulation of cancer progression remains controversial and its clinical relevance is unclear. For example, STIM1 was identified to play a potential role as a tumor growth suppressor in G401 rhabdoid tumor [14], rhabdomyosarcoma and rodent myoblast cell lines [15]. Furthermore, knockdown of STIM1 expression accelerated motility of melanoma cells, indicating that STIM1 may be an anti-metastasis gene [16]. However, more recent evidence suggests that STIM/Orai signaling accelerates migration and cell cycle progression in a number of human cancers, including breast [17], prostate [18], gastric [19] and colorectal cancer [20]. Recently, Wang *et al* [21] reported that the expression of STIM1 was significantly increased in lung cancer tissues compared with that in non-neoplastic lung tissues. Unfortunately, how STIM1 works and the mechanism of STIM1 in lung cancer is unknown.

Therefore, the purpose of the present study was to investigate the expression of the STIM1 protein in NSCLC vs. normal tissue specimens, and then perform *in vitro* and nude mouse xenograft experiments to verify the effects of STIM1 on NSCLC cells, aiming to elucidate the role of STIM1 in NSCLC cells.

## Materials and methods

### Tissue specimens

A total of 539 formalin-fixed, paraffin-embedded tissue specimens were obtained from The Department of Pathology of the Cancer Hospital of Yunnan Province, The Third Affiliated Hospital of Kunming Medical University. The specimens included 352 primary NSCLC cases and 187 cases of benign pulmonary diseases. Of the 352 NSCLC cases, 201 were adenocarcinomas and 151 were squamous cell carcinomas. The subjects included 248 male and 104 female patients, aged 33–77 years (median age, 58 years). All patients underwent surgery plus lymph node dissection. Patients with relapsed disease or those who have received radiation, chemotherapy or preoperative biotherapy were excluded from this study to avoid any changes in tumor marker determination due to the effect of the treatment. Patients diagnosed with multiple primary cancers in other organs or tissues were also excluded. Among the 187 cases with benign lung conditions, 90% were inflammatory pseudotumors, including 129 male and 58 female patients aged 16–77 years (median age, 42 years). The present study was approved by the Ethics Committee of the Third Affiliated Hospital of Kunming Medical University, and all patients provided written informed consent and authorized the use of their biological specimens for research purposes. Demographic and clinical data were obtained from the patients’ medical records.

The article "Knockdown of STIM1 expression inhibits non-small-cell lung cancer cell proliferation in vitro and in nude mouse xenografts" was published in 2019. Journal: Bioengineered.

### Immunohistochemistry

Formalin-fixed and paraffin-embedded tissue specimens were prepared for tissue microarray construction with double 3-mm core tissues of each case, and then cut into 4 μm sections for immunohistochemical analysis of STIM1 protein expression. For immunohistochemistry, the tissue microarray sections were baked at 60ºC for 2 h and then deparaffinized in xylene, followed by rehydration through a graded series of ethanols. The sections were next microwave-treated for 10 min in a citrate buffer (pH 6.0) for antigen retrieval, and then incubated in 0.3% hydrogen peroxide for 10 min to block potential endogenous peroxidase activity. Following incubation in normal serum for 30 min, the sections were incubated with a mouse monoclonal antibody against STIM1 (ab57834, Abcam, UK) at a dilution of 1:25 in phosphate-buffered saline (PBS) overnight at 4ºC. On the following day, the sections were washed three times in PBS and further incubated with a secondary antibody followed by an ABC kit (PK-4000, Vector Laboratories, USA). For color reaction, the sections were incubated briefly with 3-3ʹ-diaminobenzidine (DAB, 002941, Dako, USA.) and counterstained with hematoxylin. Human melanoma tissues were used as positive controls. For negative controls, the primary antibody was replaced with non-immunized serum. The tissues were considered to be positive for STIM1 if ≥10% of tumor cells were stained. All the tissue microarray sections were evaluated independently by three investigators who were blinded to the clinicopathological data of each case. If there was a disagreement, the tissue was again reviewed to reach a consensus.

The article "Knockdown of STIM1 expression inhibits non-small-cell lung cancer cell proliferation in vitro and in nude mouse xenografts" was published in 2019. Journal: Bioengineered.

### Cell lines and culture

A total of 11 human NSCLC cell lines were used in the present study. These lines included the adenocarcinoma H522, H2405, H2342, A549 and SPC-A-1 cell lines; the squamous cell carcinoma SW900, H1869 and SK-MES-1 cell lines; and the large-cell lung cancer H1299, H661 and H1581 cell lines. These cell lines were purchased from ATCC Bioresource Center, except for SPC-A-1, which was purchased from the Chinese Academy of Sciences Cell Bank. The cell lines were maintained in Dulbecco’s modiﬁed Eagle’s medium supplemented with 10% fetal bovine serum (10,099–141, Invitrogen, USA), 2 mM L-glutamine (21,051, Invitrogen, USA), 100 U/ml penicillin (P3032, Sigma-Aldrich, USA), and 100 mg/ml streptomycin (WB11000, Sigma-Aldrich, USA) in a humidified incubator with 5% CO_2_ at 37°C. The medium was refreshed every 2 days and cells were passaged every 2–3 days.

### Construction of lentiviral shrna vector and cell infection

To knock down STIM1 expression, a lentiviral vector carrying STIM1 shRNA was constructed using an STIM1 transcript (NM_003156, 5ʹ-CCTGGATGATGTAGATCATAA-3ʹ and 5ʹ-AGAAGGAGCUAGAAUCUCAC-3ʹ). The shRNA oligonucleotides were inserted into a pFU-GW-RNAi plasmid containing a GFP gene at the *Hpa*I and *Xho*I sites. After DNA sequence confirmation, these plasmids were named pFU-GW-STIM1-shRNA-1 (STIM1-shRNA-1) and pFU-GW-STIM1-shRNA-2 (STIM1-shRNA-2). Ascrambled lentiviral control vector, containing the same nucleotide bases but in a random order (5ʹ-TTCTCCGAACGTGTCACGT-3ʹ), was also constructed in the same manner and defined as pFU-GW-Scr-shRNA (Scr-shRNA). To produce lentivirus, 293T cells were transiently co-transfected with pFU-GW-STIM1-shRNA or pFU-GW-Scr-shRNA, together with pHelper 1.0 vector and pHelper 2.0 vector by Lipofectamine 2000 (11,668–027, Invitrogen, USA). Packaged virus was harvested from the supernatant of transfected 293T cells.

To knock down STIM1 expression, cells at 30-50% confluency were infected with STIM1-shRNAs or Scr-shRNA at a multiplicity of infection of 30 using Polybrene (5 μg/ml) overnight at 37°C. The medium was refreshed after 8–12 h. A parallel culture of cells without any treatment was used as a negative control.

### Protein extraction and western blotting

After infection with lentiviral STIM1-shRNAs or Scr-shRNA for 72 h, the cells were washed with ice-cold PBS and lysed by a 30-min incubation on ice with RIPA buffer (89,900, Pierce, USA). The cell lysate was then centrifuged at 14,000 x g, 4°C for 20 min and protein concentration was determined using the BCA assay reagent (23,227, Thermo Fisher Scientific, USA). A total of 50 μg aliquots of protein lysates were mixed with the sample buffer and boiled for 5 min, then resolved in 10% SDS-polyacrylamide gel and transferred onto a polyvinylidene fluoride membrane (ISEQ00010, EMD Millipore, USA) by electroblotting. For western blotting, the membrane was incubated in a blocking buffer (Tris-based saline containing 5% skimmed milk and 0.1% Tween 20; TBS-T) for 2 h, followed by incubation with a primary antibody against STIM1 (dilution 1:1,000) (ab57834, Abcam, UK), CDK1 and CDK2 (dilution 1:500) (ab32094, ab32147, Abcam, UK) or α-tubulin (dilution 1:1,000), (2125, Cell Signaling Technology, USA) for 16 h at 4°C. On the following day, the membrane was washed with TBS-T three times and then incubated with a specific secondary anti-mouse IgG (7076, Cell Signaling Technology, USA) or anti-rabbit IgG (7074, Cell Signaling Technology, USA) antibody conjugated with peroxidase at a dilution of 1:20,000. Relative protein intensity was detected using SuperSignal chemiluminescence system (RPN2135, GE Healthcare, USA) followed by exposure to autoradiographic film. α-tubulin was used as an internal control for equal protein loading.

The article "Knockdown of STIM1 expression inhibits non-small-cell lung cancer cell proliferation in vitro and in nude mouse xenografts" was published in 2019. Journal: Bioengineered.

### Cell growth assay

In order to assess the effect of STIM1 on NSCLC cell proliferation, A549 and SK-MES-1 cells were infected with STIM1-shRNAs or Scr-shRNA for 72 h and then harvested and seeded into 24-well plates at a density of 1.6 × 10 [4] per well for A549 cells and 2 × 10 [4] per well for SK-MES-1 cells in triplicate and grown for up to 7 days. Cells were harvested every 24 h using trypsin/EDTA and counted using an electronic cell counter (Colter Z1, Beckman Colter, Germany). All experiments were repeated three times.

### Cell viability MTS assay

Cell viability was assessed using a 3-(4,5-dimethylthiazol-2-yl)-5-(3-carboxymethoxyphenyl)-2-(4-sulfophenyl)-2H-tetrazolium (MTS) assay (G3580, Promega, USA). Briefly, A549 (4x10[3]) and SK-MES-1 (5x10[3]) cells of each group were plated into 96-well plates with 150 μl of medium and grown for up to 7 days. Six parallel wells were assigned to each group, as well as a blank control (no cells). At the end of the experiment, 30 μl of MTS substrate was added into each well and incubated for 2 h in the dark. The absorbance at 490 nm was measured using a plate reader (BMG Labtech). All experiments were performed three times independently.

### Colony formation assay

Cells at the exponential growth phase were collected from a monolayer culture through trypsinization. Approximately 200 cells were added into each well of a 6-well culture plate in triplicate and cultured in complete culture medium for 14 days. At the end of the experiment, cell colonies were washed twice with PBS, and then fixed in 100% methanol for 15–30 min and stained with Giemsa solution. The number of colonies (≥50 cells) was counted under a microscope, and colony formation was calculated relative to the number of untreated controls. The colony formation efficiency was calculated as follows: Efficiency = (number of colonies/number of cells inoculated) x 100%. Each experiment was repeated once.

The article "Knockdown of STIM1 expression inhibits non-small-cell lung cancer cell proliferation in vitro and in nude mouse xenografts" was published in 2019. Journal: Bioengineered.

### Cell cycle flow cytometry assay

The cell cycle distribution was detected by a flow cytometric analysis of DNA content. Briefly, cells were harvested by trypsin/EDTA following infection with STIM1-shRNAs or Scr-shRNA lentivirus for 48 h and washed with ice-cold PBS (pH 7.4) by centrifugation and fixed in pre-chilled 70% ethanol for at least 12 h at 4°C. The ﬁxed cells were then collected, washed three times with PBS, and suspended in PBS containing 10 *µ*g/ml propidium iodide and 100 *µ*g/ml RNase A (C1052, Beyotime Institute of Biotechnology, China), and then incubated at 37°C for at least 30 min in the dark to eliminate the intracellular RNA. DNA content was measured using a FACS Calibur system (FACS Canto^TM^ II Flow Cytometer, BD Biosciences, USA) and analyzed by Cell Quest software package for cell cycle distribution. Only signals from the single cells were included in the analysis (30,000 cells/assay). Each experiment was conducted in triplicate and repeated at least once.

### Animal experiments

The nude mouse xenograft model was constructed using 4-week-old female BALB/c nude mice. The mice were purchased from the Beijing Vital River Laboratories and were housed in pathogen-free cages (n = 5/cage) with a controlled light/dark cycle (12/12 h) at a temperature of 21°C. The animal use protocol was approved by the Institutional Animal Care Committee and all procedures conformed to Animal Studies Committee-approved protocols. Tumor xenografts were generated by subcutaneously inoculating 8x10[6] A549 cells, Scr-shRNA A549 cells, or STIM1-shRNA A549 cells in Matrigel (cat. no. 354,234, BD Biosciences)[22]. The cells were suspended in 50 μl PBS and mixed with 50 μl Matrigel, then injected into the right flank of the nude mice (5 mice per group). The tumor xenografts were measured every 3 days using a vernier caliper for the length (a) and width (b). Tumor volume (cm[3]) was calculated as follows: Volume = ab[2]/2. The mice were sacrificed 7 weeks after tumor cell inoculation, and the tumor xenografts were excised and weighed.

The article "Knockdown of STIM1 expression inhibits non-small-cell lung cancer cell proliferation in vitro and in nude mouse xenografts" was published in 2019. Journal: Bioengineered.

### Statistical analysis

The association of immunohistochemical STIM1 staining with the clinicopathological parameters of the patients was analyzed using the χ[2] test with a P-value of <0.05 considered to indicate statistically significant differences. The other data were analyzed using Student’s *t*-test, with P ≤ 0.05 considered statistically significant. All statistical analyzes were performed using SPSS v.13.0 software for Windows (SPSS Inc.).

## Results

### Differential expression of the STIM1 protein in NSCLC tissue specimens

In the present study, the expression of the STIM1 protein in 539 paraffin-embedded tissue samples was assessed. The STIM1 protein was mainly confined to the cytoplasm of epithelial cells, which exhibited 76.99% (271/352) positive staining in NSCLC cases vs. 18.72% (35/187) in benign pulmonary conditions (P = 0.00001; Figure 1(b,d)). Notably, the expression of STIM1 protein was associated with NSCLC T stage (P = 0.038). Unfortunately, no other associations with STIM1 expression were identified (Table 1).

**Table 1.** Association of STIM1 expression with clinicopathological factors in NSCLC and benign pulmonary diseases.

Clinicopathological parameter	N	STIM1-positive n (%)	*P*-value
Benign lesions	187	35 (18.72)	0.000
NSCLC	352	271 (76.99)	
Gender			
Male	248	194 (80.24)	0.394
Female	104	77 (69.23)	
Age, years			
≤65	280	215 (76.79)	0.144
>65	72	61 (84.72)	
Histology			
Squamous cell	151	110 (72.85)	0.110
Adenocarcinoma	201	161 (80.10)	
Differentiation			
High	59	47 (79.66)	0.789
Middle	214	165 (77.10)	
Low	79	59 (74.68)	
AJCC stage			
I	167	119 (71.26)	0.038
II	77	61 (79.22)	
IIIa	108	91 (84.26)	
Lymph node metastasis			
No	179	138 (77.09)	0.961
Yes	173	133 (76.88)

**Figure 1.** Expression of STIM1 in NSCLC and benign pulmonary diseases tissues. (a) Hematoxylin and eosin staining of lung adenocarcinoma. (b) Immunohistochemical staining of STIM1 protein in the cytoplasm of NSCLC cells. (c) Hematoxylin and eosin staining of tissues from a benign pulmonary disease. (d) Negative immunostaining for the STIM1 protein in a benign pulmonary disease. Scale bar: 20 μm. STIM1, stromal interaction molecule 1; NSCLC, non-small-cell lung cancer.

### Knockdown of STIM1 expression inhibits NSCLC cell proliferation

The expression of STIM1 was assessed in 11 NSCLC cell lines (i.e., H522, H2405, H2342, A549, SPC-A-1, SW900, H1869, SK-MES-1, H1299, H661 and H1581) and the STIM1 protein was found to be expressed in all those cell lines (Figure 2(a)). The expression of STIM1 in A549(adenocarcinoma) and SK-MES-1(squamous cell carcinoma) is in moderate level, so A549 and SK-MES-1 cell lines were then selected to assess knockdown of STIM1 expression and the following experiments. The cells were infected with lentivirus carrying STIM1-shRNAs or negative control shRNA (Scr-shRNA) for 3 days. Western blotting data revealed that STIM1-shRNA significantly reduced the levels of the STIM1 protein compared with Scr-shRNA-infected A549 cells (Figure 2(b)) and SK-MES-1 cells (Figure 2(c)).

The article "Knockdown of STIM1 expression inhibits non-small-cell lung cancer cell proliferation in vitro and in nude mouse xenografts" was published in 2019. Journal: Bioengineered.

**Figure 2.** Expression and knockdown of STIM1 expression in NSCLC cell lines. (a) The expressiom of STIM1 in 11 NSCLC cell lines were detected by Western blotting. (b) and (c) Western blotting analysis of STIM1 expression in A549 and SK-MES-1 cells infected with STIM1 shRNA lentivirus. α-Tubulin as used as a loading control. STIM1, stromal interaction molecule 1; NSCLC, non-small-cell lung cancer.

To determine the effect of STIM1 downregulation on the viability and proliferation of A549 and SK-MES-1 cells, cell growth assay and MTS assay were conducted. As shown in Figure 3(a), cell growth demonstrated that the growth of STIM1-shRNAs-infected cells was markedly slower compared with that of control cells (parental A549 and Scr-shRNA-infected A549 cells or parental SK-MES-1 and Scr-shRNA-infected SK-MES-1 cells). The MTS assay further confirmed this pattern of STIM1 knockdown-inhibitory effect on NSCLC cells (Figure 3(b)). Furthermore, A549 and SK-MES-1 cells with STIM1 knockdown also formed significantly fewer colonies compared with their control cells (Figure 3(c)). However, there was no significant difference between Scr-shRNA-infected cells and parental cells.

**Figure 3.** Knockdown of STIM1 inhibits cell growth and viability of NSCLC cells. (a) STIM1 knockdown significantly inhibited cell growth in A549 and SK-MES-1 cells detected by cell counting assay. (b) MTS assay detected that the viability of NSCLC cells infected STIM1-shRNA was suppressed. (c) STIM1 knockdown A549 and SK-MES-1 cells also formed significantly less colonies than those of their control cells. *p < 0.05 by Student’s t-test. STIM1, stromal interaction molecule 1. a. b. c.

### Knockdown of STIM1 expression induces A549 and SK-MES-1 cell arrest at the G2/M and s phases of the cell cycle

In order to analyze the effect of STIM1 in cell cycle, a flow cytometric assay was then conducted after knockdown of STIM1 expression. As shown in Figure 4(a), the percentage of A549 cells at the G2/M phase of the cell cycle was increased from 3.34% (parental A549 Scr-shRNA) to 6.46% or 7.64% (STIM1-shRNA-A549; P < 0.05), and the percentage of cells at the S phase of the cell cycle was increased from 11.50% to 23.89% or 21.27% (P < 0.05). By contrast, the number of G1/G0 cells was decreased (STIM1-shRNAs-A549; P < 0.05). A similar result was observed in SK-MES-1 cells (Figure 4(b)). Taken together, these ﬁndings indicate that lentivirus-mediated downregulation of STIM1 resulted in cell cycle arrest at the G2/M and S transition, which contributed to the inhibition of A549 and SK-MES-1 cell growth.

The article "Knockdown of STIM1 expression inhibits non-small-cell lung cancer cell proliferation in vitro and in nude mouse xenografts" was published in 2019. Journal: Bioengineered.

**Figure 4.** Knockdown of STIM1 expression induced cell cycle block in NSCLC cells. The cell cycle distribution was investigated in A549 and SK-MES-1 cells with STIM1 knockdown and it was observed that the S and G2/M phase population was markedly increased, while the G0/G1 phase population was significantly decreased compared with their controls. (a) Flow cytometric assay for A549 cells. (b) Flow cytometric assay for SK-MES-1 cells. *p < 0.05 by Student’s t-test. STIM1, stromal interaction molecule 1.

### Knockdown of STIM1 expression inhibits NSCLC cell proliferation through downregulation of CDK1 and CDK2 expression

To further explore the molecular events underlying the suppression of A549 and SK-MES-1 cell growth following STIM1 knockdown, the expression of CDKs was assessed using western blotting. We found that CDK1 and CDK2 were significantly downregulated after knockdown of STIM1 expression in A549 and SK-MES-1 cells (Figure 5).

**Figure 5.** Expression of cell cycle-related molecules in NSCLC cells with STIM1 knockdown. CDK1 and CDK2 were significantly downregulated after knockdown of STIM1 expression in A549 and SK-MES-1 cells. *p < 0.05 by Student’s t-test. STIM1, stromal interaction molecule 1; NSCLC, non-small-cell lung cancer.

### Knockdown of STIM1 inhibits tumorigenicity and growth of A549 cells in nude mice xenografts

To confirm the *in vitro* data, a nude mice xenograft assay was performed. For the STIM1 knockdown effect of sequence 2 is more obvious, so in the animal experiment we only use shRNA-2 to knockdown of STIM1. The data demonstrated that Matrigel substrate was completely absorbed 3 days after injection, and palpable tumors were detectable on day 7 after subcutaneous inoculation of the cells. Compared with tumor xenografts in mice implanted with A549 or Scr-shRNA-infected A549 cells, the tumor xenografts grew significantly slower following implantation of A549 STIM1-shRNA-infected cells (Figure 6(a)). Then nude mice were sacrificed 7 weeks after tumor cell inoculation and the tumors were resected and examined. On gross inspection, the tumor xenografts formed by STIM1-shRNA-infected A549 cells were markedly smaller compared with those formed by A549 or Scr-shRNA-infected A549 cells (Figure 6(b)). In addition, a significant reduction in the wet weight of tumors from STIM1-shRNA-infected tumor cell xenografts compared with the controls was observed (Figure 6(c)).

The article "Knockdown of STIM1 expression inhibits non-small-cell lung cancer cell proliferation in vitro and in nude mouse xenografts" was published in 2019. Journal: Bioengineered.

**Figure 6.** Knockdown of STIM1 expression inhibits A549 cells in nude mouse xenografts. Knockdown of STIM1 inhibited tumorigenicity and growth of A549 cells in nude mice xenografts (a) Growth curve of tumor xenografts. (b) Volume of tumor xenografts. (c) Wet weights of tumor xenografts. *P < 0.05 compared with A549 and Scr-shRNA-infected A549 cells. *p < 0.05 by Student’s t-test. STIM1, stromal interaction molecule 1; NSCLC, non-small-cell lung cancer.

## Discussion

Human carcinogenesis predominantly involves a disordered balance of cell proliferation, differentiation and apoptosis. A number of studies have provided evidence supporting that altered Ca[2]+ signaling contributes to tumorigenesis and tumor progression [23,24]. STIM1, the Ca[2]+ storage sensor protein with a single transmembrane domain localized to the ER, is the key component of SOCE. Also, STIM1 is a key activator of store-operated channels (SOCs) that allow extracellular Ca[2]+ influx into cells[25].

The present study demonstrated that STIM1 was overexpressed in NSCLC tissues and the expression of STIM1 protein was associated with advanced NSCLC T stage. Furthermore, the *in vitro* experiments demonstrated that the STIM1 protein was also expressed in all 11 human NSCLC cell lines investigated. Knockdown of STIM1 inhibited NSCLC cell proliferation *in vitro* and *in vivo*. At the molecular level, knockdown of STIM1 suppressed the expression of CDK1 and CDK2 in NSCLC cells. These data indicate that the target of the STIM1 protein may effectively control NSCLC progression.

Indeed, previous research show that the role of STIM1 in regulation of cancer progression was controversial. Some studies have suggested the STIM1 works as an oncogene. For example, downregulation of STIM1 expression inhibited glioblastoma U251 cell proliferation by inducing cell cycle arrest in the G0/G1 phase through regulation of p21^Waf^[1]/^Cip^[1], cyclin D1 and CDK4[26]. STIM1 knockdown decreased the protein levels of cyclin D1 in human cardiac c-kit^+^ progenitor cells[27]. STMI1 silencing in cervical cancer cells significantly inhibited tumor cell proliferation by arresting the cell cycle at the S and G2/M phases[28]. Knockdown of STIM1 expression enhanced NSCLC cell apoptosis induced by cisplatin[29]. However, a number of other previous studies have suggested that the STIM1 gene acts as a tumor suppressor. For example, STIM1 knockdown accelerated the motility of melanoma cells, while STIM1 overexpression induced growth arrest of G401 rhabdoid tumor[14], rhabdomyosarcoma and rodent myoblast cell lines[15]. The present *ex vivo, in vitro* and *in vivo* nude mouse data support the function of STIM1 as an oncogene, which is consistent with another lung cancer study[21]. However, further studies are required to evaluate STIM1 as a viable option in the treatment of NSCLC patients.

The article "Knockdown of STIM1 expression inhibits non-small-cell lung cancer cell proliferation in vitro and in nude mouse xenografts" was published in 2019. Journal: Bioengineered.

Furthermore, in normal cell homeostasis, STIM1 will sense and activate the ‘store-operated’ ORAI1 calcium ion channels in the plasma membrane through STIM1 EF hand domain[30]. The STIM1 protein may be phosphorylated by EKRK1/2 at Ser575, Ser608 and Ser621, and phosphorylation at all three sites is required for full interaction of the STIM1 protein with ORAI1 and activation of Ca[2]+ influx[31]. However, it is unclear whether the STIM1 protein has additional functions, such as cell proliferation and metabolic change following the alterations of cellular Ca[2]+ levels. Ca[2]+ regulates a wide array of cellular functions, including gene expression, motility and cell proliferation. SOCE, a main pathway of extracellular Ca[2]+ influx, plays a significant role in extracellular Ca[2]+ homeostasis in almost all cellular pathways[32]. SOCE is important for the regulation of contraction, cell proliferation and apoptosis, which are pathways implicated in cancer pathogenesis [33,34]. In the present study, we inhibited STIM1, the key component of SOCE, which attenuated Ca[2]+ influx and suppressed A549 and SK-MES-1 cell proliferation. Indeed, during human carcinogenesis, cancer cells overexpress STIM1 compared with normal epithelial cells[35]. A recent study investigated the role of STIM1 in tumor cell migration and the metastatic cell phenotype; increased expression of STIM1-ORAI1-based SOCE appears to promote breast cancer metastasis due to the stimulation of breast tumor cell migration[36], Furthermore, STIM1 knockdown may inhibit the invasion and migration of A549 lung cancer cells *in vitro* and *in vivo*[37]. Taken together, these findings support an oncogenic role of STIM1.

Abnormal cell proliferation caused by cell cycle dysregulation is one of the primary characteristics of cancer cells[38]. Tumor-associated cell cycle defects are often mediated by alterations in cyclins, cyclin-dependent kinases (CDKs) and CDK inhibitor (CKI) activity[39]. In the present study, knockdown of the STIM1 protein was shown to reduce the expression of CDK1 and CDK2. CDK1, also referred as cell division control protein 2, is a highly conserved protein that acts as a serine/threonine kinase, and is a key player in cell cycle regulation. CDK1 plays a critical role in the transition of cells between the G2 and M phase, as well as the execution of mitosis, and the catalytic activity of CDK1 requires B-type cyclins[40]. CDK1/cyclin B1 activity appears throughout the G2-M phase, and is turned off by cyclin B1 destruction as cells enter the anaphase of mitosis[41]. CDK2 is a catalytic subunit of the CDK complex, the activity of which is restricted to the G1-S phase of the cell cycle. Also, CDK2 has been viewed as a key cell cycle regulator that is crucial for S phase progression [42–44]. The data of the present study demonstrated that knockdown of STIM1 expression inhibited NSCLC cell proliferation by altering the cell cycle, leading to an increase in G0/G1 phase and G2/M and S phase of the cell cycle through downregulation of CDK1 and CDK2. The result was consistent with the previous study of Wang *et al*[21]. However, further studies are required to fully elucidate the molecular mechanisms underlying for the role of STIM1 in NSCLC progression.

The article "Knockdown of STIM1 expression inhibits non-small-cell lung cancer cell proliferation in vitro and in nude mouse xenografts" was published in 2019. Journal: Bioengineered.

### Practical applications and future research perspectives of this work

These data indicate that aberrant expression of the STIM1 protein may contribute to NSCLC progression. Future studies should focus on targeting STIM1 as a novel strategy for NSCLC therapy.

### Conclusion

STIM1 was highly expression in NSCLC and promoted cancer proliferation by regulating cell cycle.

## Highlights

- STIM1 was highly expressed in NSCLC tissues and correlated with T stage.
- Knocking down STIM1 inhibited NSCLC cell proliferation
- STIM1 knockdown induced NSCLC cell cycle arrest.
